The article "Monitoring of Maximum Oxygen Intake of Breathing and Heart Rate in Exercise Training Based on Regression Equations" was retracted in 2023. Reasons: signs of a paper mill; suspected computer-generated content; unreliable results or conclusions; lack of ethics approval or compliance.

# Monitoring of Maximum Oxygen Intake of Breathing and Heart Rate in Exercise Training Based on Regression Equations

**DOI:** 10.1155/2022/5025615

**Published:** 2022-03-07

**Authors:** Xiaoge Ma, Xujie Yan

**Affiliations:** ^1^School of Sports and Leisure, Guangdong Ocean University, Zhanjiang, Guangdong 524088, China; ^2^School of Physical Education Science, South China Normal University, Guangzhou, Guangdong 510631, China

## Abstract

In order to provide a new reference method and basis for the physical testing study in healthy adults aged 40∼and 49, this paper proposes a regression equation-based monitoring study of exercise training breathing and heart rate. Sixty four subjects (30 males and 34 females), aged 40∼and 49 years, were selected. First, the subjects were screened by relevant health test and medical questionnaire to exclude the subjects with exercise contraindications and high-intensity exercise; then, the incremental load test was directly measured by gas analysis, and then, the subjects who completed the maximum oxygen intake test were tested twice, the corresponding heart rate value was recorded, and walking time were averaged for calculation. We show that the regression analysis of each index yielded regression equations and cross-validation regression equations show correlation statistics for measured and inferred maximum oxygen intake of RLOOCV = 0.826 and SEELOOCV = 0.378 (L/min). The equation can effectively speculate on the maximum oxygen intake of 40∼in healthy adults aged 49, with the advantages of efficient, low cost, fast, and convenient.

## 1. Introduction

Maximum oxygen intake (VO_2max_) is the main predictor of physical activity and cardiopulmonary function, and VO_2max_ has two measurements: direct and indirect measurement [1]. The direct test method is usually done in a professional laboratory with a cardiopulmonary function detector. Because the measurement of VO_2max_ requires not only the best efforts and potential risk but also special methods and equipment, such as platform, bicycle, or gas analyzer, the direct measurement scheme of VO_2max_ is rarely applied to the common public [2]. Although the indirect assay is not accurate by direct assay, it is not need to configure expensive equipment during the test process, and the method is easy to run, suitable for measuring in a large sample population [3]. In the indirect speculation method of maximum oxygen intake, the field test generally refers to a test method of walking or running a certain distance within a given time or a given distance in the form of walking or running and then calculates the maximum oxygen intake according to relevant indicators such as heart rate, distance, and time [4].

The article "Monitoring of Maximum Oxygen Intake of Breathing and Heart Rate in Exercise Training Based on Regression Equations" was retracted in 2023. Reasons: signs of a paper mill; suspected computer-generated content; unreliable results or conclusions; lack of ethics approval or compliance.

Site test is a relatively simple and easy way to speculate on the maximum oxygen intake, especially when there is no professional equipment, and this test method is the preferred way of in-public fitness applications [5]. The reproducibility of the estimated VO_2_, based on the tertiary HR from the commuting cycle and the regression equations from test and retest, was analyzed by Id et al. Differences between the two models were also studied. For the two models, there was no significant difference between test and retest in the components of the regression equation (Y cutoff, slope, and *R* values). There were also no systematic differences in the absolute VO_2_ levels estimated between tests and retests. The relative difference between tests and retests based on estimates from three different levels of HR was 0.99 ± 11.0 (NS), 2.67 ± 6.48 (NS) and 3.57 ± 6.24% (*P* < 0.05) for 1,1.09 ± 10.6 2.75 ± 6.43 and 2.12 ± 5.92% (all NS) as model 2. However, both models have seen some large individual differences. There was no significant difference between the two models, or the estimated VO_2_ levels, in the intercept or *R* values, at the slope of the regression equation. The heart rate method showed good reproducibility at the group level, estimating oxygen consumption in the laboratory HR-VO_2_ relationship, and was based on tertiary human resources for circulating commuting [6].

Based on this study, the maximum oxygen intake of 40∼and 49 years old was established by the 1 km walking test, exploring the feasibility of walking exercise as an indirect test of adolescent heart and lung function (VO_2max_) and performing another 1 km walking test on the heart rate and physical fitness parameters as the independent variables, and the corresponding heart rate value and walking time were averaged for calculation.The relevant regression equations are obtained.The regression equation with cross validation shows a correlation statistic for measured and inferred values for maximum oxygen intake of RLOOCV = 01826 and SEELOOCV = 01378 (L/min). Using a 1 km walking test and using this equation, we can effectively speculate on the maximum oxygen intake of 40∼in healthy adults aged 49.

## 2. Research Method

### 2.1. Research Object

This experiment included 64 subjects (30 males and 34 females), aged 40∼and 49 years. Subjects were first screened by relevant health tests and medical questionnaires to exclude subjects with exercise contraindications and inability to attend high-intensity exercise and to ensure that subjects did not take medication affecting heart rate and blood pressure before performing the test.

### 2.2. Test Scheme

During the test process, the subjects first measured static indicators such as height and weight; then, the increasing load test combined with gas analysis directly measured the maximum oxygen intake; the maximum oxygen capture meter was customed EC3000 power bicycle, the starting load of 25 W, increased 25 W, per 2 min, until the maximum oxygen intake of the subject. The test gas was collected, the oxygen intake was analyzed, and the changes of blood pressure, electrocardiogram, heart rate, and other indicators were monitored. The trial was terminated if an ECG abnormality occurred during the trial (e.g., *a* > 0.2 mV decrease in the S-T segment) or a blood pressure abnormality (e.g., systolic blood pressure decreased more than 10∼20 mmHg when the load increased). The judgment criteria for the maximum oxygen intake were three indicators: (1) despite the increased output power, the oxygen intake remained unchanged or decreased; (2) HR ≧ HR_max_ (220-age); (3) respiratory quotient (RER) ≧ 1.15; (4) the subject has exerted the maximum force and was unable to maintain the specified load.

The article "Monitoring of Maximum Oxygen Intake of Breathing and Heart Rate in Exercise Training Based on Regression Equations" was retracted in 2023. Reasons: signs of a paper mill; suspected computer-generated content; unreliable results or conclusions; lack of ethics approval or compliance.

After completing the maximum oxygen dose, the subject underwent a 1 km walking test on a later day; wear a heart rate table before testing and explain the process of the test. During the test, subjects were required to walk the 1 km distance as soon as possible, and subjects were constantly encouraged to try to walk, so as to avoid subjective slack. At a distance of 1 km, immediate heart rate (sub/min) and time used for walking (min, s) were recorded and two metrics automatically were measured by the heart rate meter and recorded in the instrument. Subjects were then allowed to rest 10∼15 min, heart rate was brought to the quiet level before a second test, the same km was taken, it was recorded in the same way, and finally the index values of the two tests were averaged for calculation, namely, the average heart rate and average time of the test. The test site was on the track and field (2 and a half inner laps) or on the trail within the community where the subject lived (the distance of the trail was measured using Google Earth software).

### 2.3. Statistic Treatment

Sex, age, height, weight, BMI, walking test heart rate, and walking test time were used as independent variables (speculative variable), gender uses the virtual code (male = 1 and female = 0), stewise regression analysis was performed using the maximum oxygen intake as a dependent variable, and the data were divided into male data group, female data group, and total data group, respectively, for regression analysis; among them, the maximum oxygen intake was also divided into absolute maximum oxygen intake (L/min) and relative maximum oxygen intake (mL/kg/min) for regression analysis, respectively. Therefore, a total of data were analyzed by six different stepwise regression analyses. To obtain the corresponding regression equation, the regression equations were then cross validated using the leave-in-one method. Data that did not reach the maximum oxygen intake judgment criteria in the increasing load test were predicted using the FORECAST0 statistical function in excel software and then used for the next calculation. All data were analyzed using the microsoftexcel2003 and SPSS1710 statistical software.

The article "Monitoring of Maximum Oxygen Intake of Breathing and Heart Rate in Exercise Training Based on Regression Equations" was retracted in 2023. Reasons: signs of a paper mill; suspected computer-generated content; unreliable results or conclusions; lack of ethics approval or compliance.

## 3. Result Analysis

### 3.1. Sample Descriptive Statistical Results

Descriptive statistics of each index of subjects are shown in Table 1, where the age range is 40∼49 years, walking trial heart rate and walking trial time are the mean of heart rate and time measured in two 1 km walking trials, and maximum oxygen intake is divided into relative and absolute forms for descriptive statistics.The heart rate between men and women was basically the same, while women had longer walking trials than men and men had a greater maximum oxygen intake than women.

### 3.2. Establish Regression Equations

#### 3.2.1. Regression Equations Were Established by a Stepwise Regression Analysis

Through Table 2, we can quantitatively observe the correlation between each index and maximum oxygen intake; according to the correlation coefficient and significance level described in the table, we can see that gender for regression analysis with total sample and absolute maximum oxygen intake, as the dependent variable, is more likely to return to the model equation with better inferred accuracy. We also see in the table that the correlation between age and maximum oxygen intake is poor, which also indicates that the indicator of age may be removed out of the regression equation during performing stepwise regression analysis.

Sex, age, height, weight, BMI, walking test heart rate, and walking trial time were used as independent variables, and the virtual code (male = 1 and  = 0 female) gender used the maximum oxygen intake as the dependent variable and six gradual regression analysis of the total data, respectively, to obtain the regression equation in Table 3. The data in the observation table show the best inferred accuracy of the regression equation with the absolute maximum oxygen intake as the dependent variable in the total data group, which are as follows: maximum oxygen intake (L/min) = 61703 + 01483 × sex + 01015 × weight (kg) − 01018 × heart rate (sub/min) − 01379 × time (min).

*R* = 01851, *R*^2^ = 01724, R^2^adj = 01706, SEE = 01367 (L/min), and gender: male = 1 and female = 0.

The article "Monitoring of Maximum Oxygen Intake of Breathing and Heart Rate in Exercise Training Based on Regression Equations" was retracted in 2023. Reasons: signs of a paper mill; suspected computer-generated content; unreliable results or conclusions; lack of ethics approval or compliance.

Therefore, it is recommended to use this equation when guessing the maximum oxygen intake of 0∼9 years olds using the 1 km walking test.

#### 3.2.2. Cross-Validated Regression Equation

Using a leave-one-method cross validation of the regression equation, the corresponding RLOOCV and SEELOOCV values of the model equation, as shown in Table 3, for cross validation, partly reflect the speculative accuracy of the regression equation.  Figure 1 represents the scatter plot between the inferred maximum oxygen intake and the measured maximum oxygen intake in the regression equation recommended above.

## 4. Discussion

As can be seen in Table 3, after several stepwise regression analyses yielded five equations, the regression equation was not obtained when the male data group took the relative maximum oxygen intake as the dependent variable. The regression equation with the absolute maximum oxygen intake as the dependent variable had only the walking trial time of one independent variable. The regression equation when the absolute maximum oxygen intake was the dependent variable had three independent variables: body weight, walking trial heart rate, and walking trial time. The regression equation with the relative maximum oxygen intake as the dependent variable has two independent variables: walking trial heart rate and walking trial time. The reduced independent variable was body weight; the reason may be that the relative maximum oxygen intake is the absolute maximum oxygen intake divided by the body weight; this thus reduces the inferred contribution of body weight to the maximum oxygen intake. The regression equations in the total data group with absolute and relative maximum oxygen intake contained the four independent variables: sex, weight, walking trial heart rate, and walking trial time [7]. Although the equation for the relative maximum oxygen intake also contains the independent variable of body weight, the correlation analysis in Table 2 shows that the correlation coefficient of body weight has decreased from 0.64 to 0.12, indicating that its speculative contribution has decreased a lot. In these equations, age, height, and BMI were not included in the independent variables because the age range of subjects was limited to 40 ∼ and 49 years, and the age difference between individuals was small, so the correlation was with maximum oxygen intake, height, and BMI, which is seen in Table 2, but there are multiple collinearity problems between these two indicators, and weight was removed out of the equation during gradual regression. It can be seen below from the complex correlation coefficient *R*, determination coefficient *R*_2_, correction determination coefficient R_2_adj, and the standard error SEE of these equations. The regression equations with the absolute maximum oxygen intake were the dependent variable in the total data group. The inferred accuracy of the regression equation with the relative maximum oxygen dose as the dependent variable and the absolute maximum oxygen amount as the dependent variable was slightly worse in the female data group. The inferred accuracy of the other two regression equations is less satisfactory. Therefore, this study recommends the use of the regression equation with absolute maximum oxygen intake in the total data group as the speculative equation for applying the 1-km inferred maximum oxygen intake of 40∼49 in a walking test; this equation has already been listed in the text for [8].

The article "Monitoring of Maximum Oxygen Intake of Breathing and Heart Rate in Exercise Training Based on Regression Equations" was retracted in 2023. Reasons: signs of a paper mill; suspected computer-generated content; unreliable results or conclusions; lack of ethics approval or compliance.

The real maximum oxygen intake of this subject was calculated by indirect speculation [9]. The principle is to analyze the correlation of the data of the center rate of the experiment, fit the linear regression equations for the two indicators, and then bring the maximum heart rate calculated with the formula “maximum heart rate = 206.9–0.67 × age” into the regression equation for calculation, and the oxygen intake value is calculated as the maximum oxygen intake value of the subject. When fitting the linear regression equation between heart rate and oxygen intake, the/FORECAST0 statistical function in Microsoft Excel software functions to calculate or predict future values based on existing values [10]. This predicted value is the *y* value derived based on a given *x* value. The known values are the existing *x* value and *y* value, and then, we use linear regression to predict the new value; the specific usage can refer to Microsoft's relevant help files. So far, there is still a question of whether there is a difference between the maximum oxygen intake calculated by this prediction method and that actually measured. To test this hypothesis, the data reaching the maximum oxygen intake measurement criterion were calculated using the same prediction method; then, the calculated maximum oxygen intake data and measured data were paired by *t*-test to test the difference between them, which showed *P* = 0.162 > 0.05 (*n* = 50), indicating no significant difference.That is, the maximum oxygen intake data calculated in this speculative way still have a certain reliability, and these data can be used to conduct the next statistical analysis.

## 5. Conclusions

In conclusion, this study established a regression equation by obtaining the heart rate at the end of walking and the gender, age, height, and weight.The regression equation can effectively speculate the maximum oxygen intake of 40∼healthy adults aged 49 and establish a site test scheme with the level of Chinese cardiopulmonary function as the standard. This new indirect test method has the advantages of high efficiency, low cost, fast, and convenient and is of important significance for guiding public scientific fitness.

The article "Monitoring of Maximum Oxygen Intake of Breathing and Heart Rate in Exercise Training Based on Regression Equations" was retracted in 2023. Reasons: signs of a paper mill; suspected computer-generated content; unreliable results or conclusions; lack of ethics approval or compliance.

## Figures and Tables

**Figure 1:** Scatter plot between inferred maximum oxygen intake and measured maximum oxygen intake in Figure 1 (*n* = 64).

**Table 1:** Descriptive statistics of each item of the subject $\left(\bar{X}\pm s\right)$.

Index	Male (*n* = 30)	Female (*n* = 34)	Total (*n* = 64)
Age (year)	44.5 ± 3.2	44.9 ± 2.7	44.8 ± 2.9
Height (cm)	171.3 ± 4.7	160.2 ± 6.3	165.4 ± 7.9
Weight (kg)	76.6 ± 11.8	62.4 ± 9.9	69.0 ± 12.9
BMI (kg·m^−1^)	26.0 ± 3.5	24.3 ± 3.3	25.1 ± 3.5
Walking trial heart rate·(sub-min^−1^)	125 ± 11	125 ± 11	125 ± 11
Time of the walking test (min)	9.37 ± 0.64	9.97 ± 0.47	9.669 ± 0.63
Absolute maximum oxygen intake (L·min^−1^)	2.58 ± 0.59	1.65 ± 0.40	2.08 ± 0.68
Relative maximum oxygen intake (mL·kg^−1^·min^−1^)	33.8 ± 7.1	26.7 ± 5.2	30.1 ± 7.1

**Table 2:** Analysis of maximum oxygen intake and other indicators.

Index	Male (*n* = 30)		Female (*n* = 34)		Total (*n* = 64)	
	Opposite VO_2max_	Absolute VO_2max_	Opposite VO_2max_	Absolute VO_2max_	Opposite VO_2max_	Absolute VO_2max_
Sex	—	—	—	—	0.69^∗∗^	0.50^∗∗^
Age (year)	0.23	0.33^*∗*^	0.16	0.02	0.10	0.14
Height (cm)	0.22	−0.19	0.37^*∗*^	−0.02	0.63^∗∗∗^	0.30^∗∗^
Weight (kg)	0.35^*∗*^	−0.27	0.54^∗∗∗^	−0.13	0.64^∗∗∗^	0.12
BMI (kg·m^−1^)	0.34^*∗*^	−0.24	0.42^∗∗^	−0.15	0.43^∗∗∗^	−0.04
Walking trial of heart rate/session·(min^−1^)	−0.29	−0.30	−0.50^∗∗^	−0.45^∗∗^	−0.27^∗∗^	−0.32^∗∗^
Time of the walking test (min)	−0.51^∗∗^	−0.36^*∗*^	−0.27	−0.29^*∗*^	−0.60^∗∗∗^	−0.49^∗∗∗^

^*∗*^ *P* < 0.05, ^∗∗^*P* < 0.01, and ^∗∗∗^*P* < 0.001. The other tables are the same.

**Table 3:** One kilometer walk test speculation maximum oxygen content regression equation.

Index	Male (*n* = 30)		Female (*n* = 34)		Total (*n* = 64)	
	Opposite VO_2max_	Absolute VO_2max_	Opposite VO_2max_	Absolute VO_2max_	Opposite VO_2max_	Absolute VO_2max_
*Equation statistic*						
Intercept	6.956	—	6.225	106.751	6.703	116.081
Sex	—	—	—	—	0.483	6.671
Age (year)	—	—	—	—	—	—
Height (cm)	—	—	—	—	—	—
Weight (kg)	—	—	−0.018	—	0.015	−0.175
BMI (kg·m^−1^)	—	—	—	—	—	—
Walking trial of heart rate/session·(min^−1^)	—	—	−0.018	−0.257	−0.018	−0.243
Walking test time (min)	−0.467	—	−0.346	−4.794	−0.379	−4.813
R	0.509	—	0.784	0.613	0.851	0.727
*R* ^2^	0.259	—	0.615	0.376	0.724	0.528
R^2^adj	0.232	—	0.577	0.336	0.706	0.493
SEE	0.513	—	0.258	4.27	0.367	5.05

*Equation test statistics*						
Durbin–Watson	2.047	—	2.094	1.957	1.889	1.868
Tolerance (minimum value)	1.000	—	0.906	0.938	0.605	0.605
VIF (maximal value)	1.000	—	1.104	1.066	1.653	1.653
*P* test for standard residues	0.994	—	0.804	0.911	0.898	0.989

*Cross-validation statistic*						
RLOOCV	0.419	—	0.711	0.509	0.826	0.678
SEELOOCV	0.525	—	0.276	4.47	0.378	5.20

The article "Monitoring of Maximum Oxygen Intake of Breathing and Heart Rate in Exercise Training Based on Regression Equations" was retracted in 2023. Reasons: signs of a paper mill; suspected computer-generated content; unreliable results or conclusions; lack of ethics approval or compliance.

## Data Availability

The data used to support the findings of this study are available from the corresponding author upon request.
